# Large-Scale Customized Production Scheduling of Multiagent-Based Medical 3D Printing

**DOI:** 10.1155/2022/6557137

**Published:** 2022-07-18

**Authors:** Jianjia He, Jian Wu, Ye Zhang, Yaopeng Wang, Hua He

**Affiliations:** ^1^Business School, University of Shanghai for Science and Technology, Shanghai 200093, China; ^2^Supper Network Research Centre (China), University of Shanghai for Science and Technology, Shanghai 200093, China; ^3^Dept of Biobank, Shanghai Chest Hospital, Shanghai Jiaotong University, Shanghai 200030, China; ^4^Department of Neurosurgery, Third Affiliated Hospital, Naval Medical University, Shanghai 200438, China

## Abstract

Three-dimensional (3D) printing, also known as additive manufacturing, has unique advantages over traditional manufacturing technologies; thus, it has attracted widespread attention in the medical field. Especially in the context of the frequent occurrence of major public health events, where the medical industry's demand for large-scale and customized production is increasing, traditional 3D printing production scheduling methods take a long time to handle large-scale customized medical 3D printing (M-3DP) production and have weak intelligent collaboration ability in the face of job-to-device matching under multimaterial printing. Given the problem caused by M-3DP large-scale customized production scheduling, an intelligent collaborative scheduling multiagent-based method is proposed in this study. First, a multiagent-based optimization model is established. On this basis, an improved genetic algorithm embedded with the product mix strategy and the intelligent matching mechanism is designed to optimize the completion time and load balance between devices. Finally, the effectiveness of the proposed method is evaluated using numerical simulation. The simulation results indicated that compared with the simple genetic algorithm, particle swarm optimization, and snake optimizer, the improved genetic algorithm could better reduce the M-3DP mass customization production scheduling time, optimize the load balance between devices, and promote the “intelligent manufacturing” process of M-3DP mass customization.

## 1. Introduction

Medical three-dimensional printing (M-3DP) is an interdisciplinary and cutting-edge emerging technology that integrates additive manufacturing, medicine, and material science. It realizes the need for personalized customization and the ground-breaking transformation from subtractive manufacturing to additive manufacturing, which reduces the development cycle and cost of products. M-3DP technology has the advantage of high digitization, rapid prototyping, and product customization [1], which is already applied to surgical planning, revision surgery, and other medical purposes [2]. With the frequent occurrence of major public health events in the world and the increasing demand for large-scale and customized production of medical products [3], M-3DP technology has been improved, while facing increased requirements placed on its large-scale customized production scheduling capability. However, few researchers have considered the product allocation and production scheduling in 3D printing (3DP) from the perspective of large-scale customized production and multi-printing materials.

At present, most studies focus on 3D printing allocation and production scheduling under a single printing material that has already been discussed from different perspectives. To clarify the research status in the field of 3D printing production scheduling, a comprehensive taxonomy covering 3DP allocation and scheduling problems is proposed (Figure 1), which is based on a hierarchy of general literature and consists of four parts: 3DP devices, material, methodology, and optimization goals. From the perspective of 3DP devices, researchers have studied the situations of machines with the same or different specifications [4, 5] and of single or multiple machines [5–9]. From the perspective of printing materials, Rohaninejad et al. [9] discussed the scheduling optimization problem of different parallel laser melting devices when producing parts with different printing materials. Li et al. [4] studied the scheduling cost optimization problem for different parallel devices with a single material. From the perspective of methodology, since the 3DP workshop scheduling problem is an NP-hard problem with no fixed solution, different scholars have adopted different methods in the research on 3D printing scheduling. Wu et al. [10] and Kucukkoc [6] adopted mixed-integer linear programming and a heuristic algorithm to optimize the scheduling problem in different situations. Zhou et al. [11] established a task matching and scheduling model for distributed 3DP services in a cloud manufacturing environment and obtained the optimal solution by improving the genetic algorithm (GA). De Antón et al. [12] used the combinatorial auction and heuristic algorithm to solve the allocation problem of 3DP parts. Rohaninejad et al. [9] constructed a biobjective mathematical model targeting makespan and the total tardiness penalty and developed an efficient hybrid meta-heuristic algorithm to solve the production shop scheduling problem under heterogeneous 3D printing equipment. Che et al. [13] established a mixed-integer linear programming model and applied a simulated annealing algorithm with designed packing strategies based on the skyline representation of packing pattern to solve the problem of machine scheduling with orientation selection and two-dimensional packing in a 3D production workshop. Based on extensive literature research, it was found that because the intelligent optimization algorithm is not constrained by specific problems, it is widely used in the field of production workshop scheduling by imitating the biological evolution of nature [14–16]. Different intelligent optimization algorithms were adopted by researchers in the heuristic algorithms, including GA [3, 7, 11, 17], particle swarm optimization (PSO) [17], and water wave optimization algorithm [16]. Moreover, some researchers have compared GA, PSO, and other heuristic algorithms and found that GA is widely used in 3D printing shop scheduling problems because of its good robustness and global optimization ability compared with other algorithms [17]. Simultaneously, the GA was found to have the strong capability and high stability in processing parallel tasks [18], making it suitable for solving the production scheduling model including multiple parallel tasks. Therefore, this study attempts to develop an improved genetic algorithm (IGA) to solve the 3D printing shop scheduling problem. From the perspective of optimization goals, existing studies have focused on the minimization of cost or the maximization of profit [4, 8, 10, 12, 19], minimization of maximum completion time [2, 6–8, 14, 15], and minimization of total energy consumption [14].

With the continuous development of professional 3DP devices and medical printing materials, M-3DP large-scale customized production has become a reality. At the treatment stage, 3D printers are under investigation for the concept of personalized medicine by allowing patients access to on-demand, customizable therapeutics [20]. Tuomi et al. [21] believed that the medial application of 3DP was mainly in the fields of tissue engineering, preoperative planning, inert implants, orthodontic treatment, postoperative support structures, and surgical instruments. In addition, with the frequent occurrence of major international public health events, such as during the COVID-19 pandemic, diverse health systems around the world were overloaded, and supply chains were disrupted due to excessive numbers of patients, resulting in shortages of medical devices and personal protective equipment [22], while 3DP can effectively prevent equipment shortages and supply chain disruptions from recurring. Therefore, it is particularly important to formulate effective large-scale production scheduling methods for M-3DP. However, there are currently few studies on M-3DP large-scale customized production scheduling. The materials of M-3DP are diverse, and the intelligent collaboration of devices and jobs needs to be considered in large-scale customized production. Therefore, the traditional 3DP production scheduling methods fail to support M-3DP, showing incapability in the face of intelligent collaborative production scheduling with multiple parallel tasks. It is urgently needed to find a new method to realize M-3DP large-scale customized production.

In view of the above, a multiagent-based M-3DP large-scale customized production scheduling method is proposed, which divides all the products in the order list into different tasks according to the reclassification rule. On this basis, a multiagent-based optimization model is established, which is solved using the improved GA to obtain the minimum order completion time and optimal load balance between devices. Finally, numerical simulation is conducted to verify the effectiveness and rationality of the proposed method.

## 2. Problem Description

Compared with 3DP of single material production, the production scheduling of M-3DP is different. Taking the stereo light curing process as an example, the main differences are as follows: since the liquid tank of the device can only be filled with one type of material at the same time, products of different materials cannot be placed in the same job for production, and material replacement is required if the material types of two serially produced jobs on one device are different. Also, compared with the traditional batch scheduling problem, the processable capacity in the task set division process is not a simple one-dimensional knapsack problem, but a more complex irregular rectangular discharge problem. Taking the projected area of the medical product layering direction as the emission basis, ensuring a certain gap between products, and making full use of the equipment processing platform have a significant impact on the order completion time. Therefore, to shorten the order completion time, a problem arises due to the irregular arrangement of different medical products on the two-dimensional (2D) plane according to their materials, heights, and shapes, i.e., the problem of task set division. Also, some products cannot be allocated to certain 3DP devices due to the limitations on capacity and maximum support height. And the load balance between devices needs to be considered when matching devices and jobs. Consequently, to reduce the load deviation between devices and shorten the order completion time, the problem of intelligent matching between jobs and devices arises. Task sets division problem and job-to-device intelligent matching problem are typical NP-hard problems, 3DP shop scheduling problem as a combination of the two, coupled with the special process of 3DP, is also an NP-hard problem.

In the case study, medical product set **I** is required to be produced on 3DP devices, and these medical products have different requirements for printing material, volume, and height. First, all medical products were assigned to different task sets according to the reclassification rule which was based on the printing material. Subsequently, each task set was divided into jobs according to the product mix strategy, which was intelligently matched to the corresponding 3DP devices. Since the task set division process and job-to-device matching process required intelligent coordination, multiagent collaboration was adopted by converting the different entities such as the 3DP devices, medical products, and jobs into agents, which could be intelligently coordinated and controlled for production, at the same time to design an improved genetic algorithm is to divide and matching for the integrated execution. This paper combined the task set division problem in M-3DP large-scale customized production with the job-to-device matching problem to optimize the total production time and load balance between devices.  Figure 2 shows a simplified flow chart of the M-3DP large-scale customized production scheduling process.

## 3. Multiagent Optimization Model

### 3.1. Assumption Setting

1. All products in the order list did not have a size exceeding the maximum constraints of the size of the printing platform.
2. Products with the same printing materials could be arbitrarily allocated in one job, whereas products of different printing materials could not be produced in the same job.
3. All products to be processed were arranged at a spacing of 10 mm to prevent the products from coming into contact and becoming damaged during the production process.
4. 3DP devices could process multiple medical products simultaneously, but new products could not be added during the job production, and the ongoing processing of the 3DP customized products could not be stopped either; the probability of printing each product successfully was 100%.
5. The length, width, height, and layering direction of each product were known in advance, and each product was arranged according to the 2D projection along the layering direction without any overlap between products allowed.

### 3.2. Symbolic Variable Description

#### 3.2.1. Set Variables and Indexes

**I** represented the set of medical products, *i* ∈ *I*, where *i* is the index of medical products.

**R** represented the task set, *r* ∈ *R*, where *r* is the index of tasks.

**M** represented the set of 3DP devices, *m* ∈ *M*, where *m* is the index of devices.

**J** represented the set of jobs, *j* ∈ *J*, where *j* is the index of jobs.

#### 3.2.2. Relevant Parameters

*T*_*mj*_ denoted the total production time to complete *j* jobs on the *m*th 3D printing device.

*C*_*mj*_ denoted the total time cost to complete the *j*-th job on the *m*th 3D printing device.

*C*_*mis*_ denoted the scanning time for the *i*th medical product on the *m*th 3D printing device.

*C*_*mij*_ denoted the processing time for the *i*th medical product on the *m*th 3D printing device.

*C*_*mjs*_ denoted the scanning time for the *j*th job on the *m*th 3D printing device.

*C*_*mjj*_ denoted the processing time for the *j*th job on the *m*th 3D printing device.

*C*_*mp*_ denoted the preparation time before the job production of the *m*th 3D printing device, value: [30:90] min.

*C*_*ma*_ denoted the processing time after the job production of the *m*th 3D printing device, value: [30:90] min.

*C*_*me*_ denoted the time it takes to replace the printing material on the *m*th 3D printing device, value: 180 min;

*F* denoted the standard deviation of the load of the 3D printing devices;

*a*_*i*_ denoted the projected area of medical product *i*;

*A*_*m*_ denoted the total area of the processing platform of the *m*th 3D printing device.

*E*_*i*_ denoted the material type of medical product *i.*

*x*_*o*_, *y*_*o*_, *z*_*o*_ denoted the coordinates of the *o*th point of the medical products.

*x*_min_, *y*_min_, *z*_min_ denoted the minimum coordinates of the 3DP devices in the three-dimensional coordinate system.

*L*_*m*_, *W*_*m*_, *H*_*m*_ denoted the length, width, and height of the processing platform of *m*th 3DP devices, respectively.

*l*_*i*_, *w*_*i*_, *h*_*i*_ denoted the length, width, and height of the *i*th medical product, respectively.

#### 3.2.3. Decision-Making Variable

(1) $$\begin{array}{c} X_{mji}=\left\{\begin{array}{cc} 1 & \text{product }i\text{ is processed in job }j\text{ by device }m\\ 0 & \text{Otherwise.} \end{array}\right.\\ L_{mj_{1}j_{2}}=\left\{\begin{array}{cc} 1 & \text{jobs }j_{1}\text{ and }j_{2}\text{ are printed continuously by device }m,\\ 0 & \text{Otherwise.} \end{array}\right.\\ D_{j_{1}j_{2}}=\left\{\begin{array}{cc} 1 & \text{jobs }j_{1}\text{ and}j_{2}\text{ have different printing materials,}\\ 0 & \text{Otherwise.} \end{array}\right. \end{array}$$

### 3.3. Objective Function Setting

Considering patients' urgent needs for medical products, the objective function minimizes the makespan of the ordered products.

(2) $$\begin{array}{c} \text{min}T=\text{max}\left(T_{mj}\right). \end{array}$$

### 3.4. Constraint Condition Establishment

The constraint conditions of the mathematical model came from stereo lithography appearance (SLA) printing process constraints and 3DP production scheduling rules, so the following constraints were established:

(3) $$\begin{array}{c} \sum_{m\in M}\sum_{j\in J}X_{mji}=1;\;\forall i\in I, \end{array}$$

(4) $$\begin{array}{c} x_{\min}\leq x_{o}\leq x_{\min}+W;\forall o\in i,\forall i\in I, \end{array}$$

(5) $$\begin{array}{c} y_{\min}\leq y_{o}\leq y_{\min}+V;\forall o\in i,\forall i\in I, \end{array}$$

(6) $$\begin{array}{c} z_{\min}\leq z_{o}\leq z_{\min}+H;\forall o\in i,\forall i\in I, \end{array}$$

(7) $$\begin{array}{c} A_{m}\geq \sum_{i\in I}X_{mji}x_{i}y_{i};\forall j\in J,\forall m\in M, \end{array}$$

(8) $$\begin{array}{c} P_{i1}\cap P_{i2}=\emptyset ,\forall i_{1},i_{2}\in I,i_{1}\neq i_{2}. \end{array}$$

Equation (3) ensures that each product is assigned to a job and produced by a 3DP device. Equations (4) through (6) indicated that all products had to be arranged on the processing platform of the 3DP devices. Equation (7) ensured that the total area of products allocated to the same job was smaller than the area of the processing platform of the 3DP device. Equation (8) ensured that there was no overlap between products.

(9) $$\begin{array}{c} C_{me}=180\sum_{j_{1}\in J}\sum_{j_{2}\in J}L_{mj_{1}j_{2}}D_{j_{1}j_{2}};j_{1}\neq j_{2},m\in M, \end{array}$$

(10) $$\begin{array}{c} T_{mj}\geq \sum_{j\in J}C_{mj};\forall m\in M, \end{array}$$

(11) $$\begin{array}{c} T_{mj}=\left\{\begin{array}{cc} C_{mj}, & j=1,\\ T_{m\left(j-1\right)}+C_{mj}+C_{me}, & j>1, \end{array}\right. \end{array}$$

(12) $$\begin{array}{c} C_{j}=C_{p}+C_{mjs}+C_{mjj}+C_{a}, \end{array}$$

(13) $$\begin{array}{c} C_{mjs}=\sum_{i\in I}X_{mji}C_{mis},\forall j\in J,\forall m\in M, \end{array}$$

(14) $$\begin{array}{c} C_{mjj}=\max\left(X_{mji}C_{mij}\right),\forall i\in I,\forall j\in J,\forall m\in M. \end{array}$$

Equation (9) is used to calculate the time for the *m*th device to replace the printing material. Equation (10) was the minimized completion time to print a job. Equation (11) represented the total production time of the device *m* when the requirement to be produced by device *m* consisted of a single job or multiple jobs. Equation (12) was the total time cost per job estimated based on the SLA printing process. The calculation considered preparation time, scanning time, processing time, and postprocessing time, where the scanning time was dependent on the area to be printed per layer, the processing time was dependent on the height of the products, and preparation time and postprocessing time consisted of material preparation, filling of protective gas, preheating, and postcooling of printing materials. Since the SLA printing was layer by layer; i.e., the laser beam scanned each product in each layer one by one, the scanning time of a job could be simplified to the sum of the scanning time of all products in the job, as shown in Equation (13). Moreover, the processing time during SLA printing was determined by the layer changing time, and it was known that layer changing occurred for all the products in the same job. The processing time of a job was determined by the product with the longest processing time in the job, as shown in Equation (14).

(15) $$\begin{array}{c} L\left(m\right)=\sum_{j\in J}C_{mj}, \end{array}$$

(16) $$\begin{array}{c} F=\sqrt{\frac{1}{n}\sum_{m\in M}{\left(L\left(m\right)-avgL\left(m\right)\right)}^{2}}. \end{array}$$

To keep the 3DP devices in a relatively good production state and shorten the printing time, a load balancing constraint was established. Equation (15) defined the total production time of the *m*th 3DP devices as its load, Equation (16) represented the overall load balance of the 3DP devices, with *F* being the standard deviation.

## 4. Improved GA Design

To optimize the production scheme of the above 3DP shop scheduling problem, this paper proposes an improved genetic algorithm (IGA). IGA combines genetic algorithms with heuristic optimization rules that take into account SLA production characteristics and product discharge issues, while solving the problem of task set division and allocating jobs to different devices in scheduling. The flow of the IGA is shown in Figure 3. The main steps are as follows: First, according to the medical product to be printed, use the initialization strategy to generate an initialization population, and then repeat the evaluation, selection, crossover, and mutation until the termination criteria are met. Among them, the calculation of the fitness value of each individual mainly includes three steps: first, to realize the arrangement of medical product positions; second, to realize the matching between jobs and devices; third, to calculate the completion time of the order according to the arrangement and matching results time.

### 4.1. Coding

Integer coding was adopted for the task sets division process and intelligent matching process, as shown in Table 1. Each row represents the medical products contained in a task, corresponding to different product agents. By changing the order of the products in any task set, new coding results were generated.

### 4.2. Initialization Selection

Most existing studies used random initialization methods, which could not guarantee the quality of the initialized population, and it was time-consuming to find the optimal solution. It was known from previous studies that mass production of products of similar height could improve production efficiency. Simultaneously, a highly-random initialization method was used for the tasks to ensure the diversity of the initial population; i.e.,10% of the chromosome sequences were obtained by the first-fit decreasing sorting algorithm, and the rest of the chromosomes were randomly generated, to study the problem of task sets division and intelligent matching.

### 4.3. Fitness Calculation

Firstly, the chromosomes were decoded, and the task sets were divided into jobs by the lowest horizontal line method according to the sequence after decoding. After obtaining the jobs, the completion time of each job was calculated according to equation (12). Secondly, the device agent and the job agent are intelligently coordinated through the intelligent matching mechanism (IMM), and then the total processing time of the order was calculated using equation (11). Finally, Equation (17) was used to calculate the fitness of the population, where *F*_*ina*_ denoted the fitness of the *a*th individual, *T*_max_ denoted the maximum total production time of the current generation population, and *T*_*ina*_ denoted the order production time for the *a*th individual.

(17) $$\begin{array}{c} F_{ina}=1.1\times T_{\max}-T_{ina}. \end{array}$$

#### 4.3.1. Product Mix Strategy

In view of the product mix strategy, an improved lowest horizontal line method is designed (Figure 4), which is mainly improved from two aspects. First of all, a plus and minus sign is randomly added to the gene during encoding, so there is a plus and minus sign in the decoded sequence. The plus sign indicates that the product does not rotate 90° and is directly placed into the processing platform according to the rules, while the minus sign is the opposite. Secondly, the product will be rotated by 90° during the arrangement process if the product cannot be placed in the lowest horizontal line before the merger, and then judged whether it can be placed again. Such improvements can expand the optimization space of the GA to obtain better arrangement results, thereby improving the utilization of processing platforms and shortening the completion time of orders. The specific steps of this method are as follows:

  Step 1 Initialize the lowest horizontal line set (Line), which only includes Line_**0**_ = (0, *W*_*m*_, 0).
  Step 2 In terms of the decoded sequence order, the next medical product *i* to be arranged is selected. First, judge whether to rotate the product *i* according to the sign and then inquire whether there is Line_i_ with *a* width greater than *w*_*i*_ and the lowest height in Line. If it exists (see Figure 4(a)), go to Step 3; If it does not exist (see Figure 4(b)), rotate the product *i* by 90°, and then re-query whether there is Line_i_ with a width greater than *l*_i_ and the lowest height in Line. If it exists (see Figure 4(c)), go to Step 3; If it still does not exist after rotation (see Figure 4(d)), go to Step 4.
  Step 3 Arrange product *i* into the leftmost end of Line_*i*_, update the Line, and go to Step 5.
  Step 4 Select a horizontal line with a lower height adjacent to the lowest horizontal line, raise the lowest horizontal line to be flush with the horizontal line (see Figure 4(e)), update Line, and go to Step 2.
  Step 5 Determine whether all medical products have been arranged. If the arrangement is complete, end, otherwise go to Step 2.

#### 4.3.2. Intelligent Matching Mechanism

In view of the intelligent matching process between jobs and 3DP device resources, a multiagent intelligent matching mechanism was established (Figure 5), including the resource layer that stored the status of 3DP devices and the task layer that stored job information. Simultaneously, a management layer was set up to complete the information exchange between the resource and task layers to achieve intelligent matching between jobs and 3DP devices. Also, the function of the managing agent was to control, supervise, and coordinate the execution process of each agent in the model. Each 3DP device agent corresponded to the 3DP devices fed back the device status information to the managing agent in real time and accepted the scheduling of the managing agent. Each job agent corresponded to the job sent the information including production time and printing materials required for each job to the managing agent in real time and accepted the assignment of the managing agent. Each job agent had an equal probability to be matched to any 3DP device agent, and the optimal matching results were given based on the decision-making condition. This mechanism could improve the matching capability with multiple resources and multiple tasks in the intelligent cooperative scheduling problem and optimize the load balance among 3DP devices.

IMM mainly includes two important processes: task requirements and resource matching. During the task requirement setup process, the job *j* submitted task condition limits to the managing agent and applied for resource *m*, and the task condition limiting vector was **Y**_**n**_ = (*C*_*mj*_, *E*, max(*l*_*i*_), max(*w*_*i*_), max(*h*_*i*_)), where *C*_*mj*_ denoted the total time cost to complete the *j*th job on the *m*th 3D printing device; *E* denoted the material type of the job; max(*l*_*i*_), max(*w*_*i*_), max(*h*_*i*_) represented the largest length, width, and height of products in the same job, respectively. The above data was stored in the dynamic information database. During the resource matching process, the jobs were arranged in descending order of production time, then matched with the 3DP devices one by one according to the matching rules. The managing agent received the task condition limiting vector **Y**_**n**_, forwarded it to each device in the resource layer, and queried the dynamic information databases for 3DP devices that satisfied the data variables *L* ≥ max(*l*_*i*_), *W* ≥ max(*w*_*i*_), and *H* ≥ max(*h*_*i*_). If such **M** was unavailable, a message indicating the job could not be completed was returned. Otherwise, it again queried the dynamic information database for the 3DP devices with the lowest working load as the output device, which was returned to the managing agent. Also, if the printing material for the previous job was different from that for the following job, additional time for changing the printing materials became necessary.

### 4.4. Selection

In the selection process, a strategy combining roulette selection and elite selection was proposed to overcome the slow convergence speed of GA in processing parallel tasks. The selection probability of an individual was based on equation (18), where *P*_*ina*_ denoted the probability of selecting *a*th individual in the population, and *e* denoted the population size of each generation.

(18) $$\begin{array}{c} P_{ina}=\frac{F_{ina}}{\sum_{a=1}^{e}F_{ina}}. \end{array}$$

### 4.5. Crossover and Mutation

To improve the crossover efficiency of the population, a product sequence-based crossover method was adopted to change the product arrangement during processing. Assuming *P*_1_ and *P*_2_ were two-parent generations, the crossover was as follows:

(1) All products were randomly divided into either *S*_1_ or *S*_2_, where *S*_1_ denoted the first set of products and S_2_ denoted the second set of products.
  (19) $$\begin{array}{c} P_{1}=\left[\begin{array}{ccccc} 5 & 4 & 2 & 1 & 3 \end{array}\right]P_{2}=\left[\begin{array}{ccccc} 2 & 4 & 3 & 1 & 5 \end{array}\right],\\ S_{1}=\left[\begin{array}{ccc} 1 & 3 & 4 \end{array}\right]S_{2}=\left[\begin{array}{cc} 2 & 5 \end{array}\right]. \end{array}$$
(2) The product sequences belonging to *S*_1_(*S*_2_) in *P*_1_(*P*_2_) were copied to *D*_1_(*D*_2_).
  (20) $$\begin{array}{c} D_{1}=\left[\begin{array}{ccccc} . & 4 & . & 1 & 3 \end{array}\right]D_{2}=\left[\begin{array}{ccc} 1 & \ldots & 5 \end{array}\right]. \end{array}$$
(3) The product sequences belonging to *S*_1_(*S*_2_) in *P*_1_(*P*_2_) were copied to *D*_2_(*D*_1_). The chromosomes of the two descendent generations after crossover were respectively:
  (21) $$\begin{array}{c} D_{1}=\left[\begin{array}{ccccc} 2 & 4 & 5 & 3 & 1 \end{array}\right]D_{2}=\left[\begin{array}{ccccc} 2 & 4 & 1 & 3 & 5 \end{array}\right]. \end{array}$$

Also, chromosomal mutation conventionally referred to the random mutation of genes in the chromosomes, which would lead to repeated production or missed production of products. Therefore, the method of exchanging genes was adopted; i.e., two genes in a chromosome were selected to be exchanged in sequence. Assuming *P*_1_ was a parent generation, the mutation was as follows:

(1) Two genes were randomly selected from the parent generation *P*_1_ into *S*_1_.
  (22) $$\begin{array}{c} P_{1}=\left[\begin{array}{ccccc} 5 & 4 & 2 & 1 & 3 \end{array}\right]S_{1}=\left[\begin{array}{cc} 5 & 2 \end{array}\right]. \end{array}$$
(2) The positions of the two genes in *S*_1_ were exchanged in the parent generation *P*_1_, so that the descendent generation had the following chromosomes after mutation:
  (23) $$\begin{array}{c} D_{1}=\left[\begin{array}{ccccc} 2 & 4 & 5 & 1 & 3 \end{array}\right]. \end{array}$$

## 5. Results and Discussion

### 5.1. Experiment Design

Since there were many 3DP processes, it was difficult to find available experimental results for direct comparison. Moreover, since the 3DP production was slow, it was time-consuming and costly to conduct various comparative experiments. Therefore, numerical simulation was used to verify the proposed M-3DP large-scale customized production scheduling method. In terms of the selection of medical products, the medical product models were downloaded from relevant websites, which were used as a customized 3DP production order list for a certain hospital. There were 70 products in the order list, including tissue and organ models required for preoperative simulation, prosthetics, splints, medical tools, and auxiliary devices. In terms of the selection of printing materials, since there were many types of printing materials for M-3DP, the production scheduling of medical products with two different types of printing materials was studied to ensure that the experimental results were more comprehensive. In terms of the selection of printing devices, since SLA technology had significant advantages in mass production, precision manufacturing, and customized manufacturing, and was widely used by major manufacturers, the LT450 was selected as the device. It was assumed that all the products had no special performance requirements so that they could all be produced by the LT450 device. The support for each product was generated through the Materialise Magics 24.0 software based on the device parameters of LT450, and the scanning time and processing time of each product were estimated.  Table 2 shows the specific data. Also, to verify the processing capability of the proposed method in different scenarios, the experimental scenarios are set as follows: 70 medical products and two to eight sets of 3DP devices. The ability of intelligent collaborative scheduling method to optimize processing time and device load balancing under different production resources were studied.

### 5.2. Experimental Results and Discussion

To verify the applicability of the genetic algorithm compared with other algorithms in processing 3DP workshop scheduling, the PSO and the snake optimizer (SO) with the IMM were designed respectively, and the optimization capabilities of each algorithm for shortening the order completion time and devices load balancing were compared. In Table 3, the same number of iterations, population size, and corresponding parameters are set for each algorithm.

Each algorithm runs under the corresponding parameter settings, and the obtained minimum order completion time and device load standard deviation are shown in Table 4. The data in brackets represent the load standard deviation of devices under the current scenario, and the data outside the brackets represent the minimum order completion time under the current scenario. It can be concluded from the table that IGA outperforms other algorithms in all scenarios and has better solution quality. This is because the crossover mutation of IGA is more suitable for the 3D printing shop scheduling problem when the population is updated and iterative, while the PSO often repeats or misses the number of a certain dimension when updating the particle position, which will lead to the global search ability deviation in later modification. The SO can be regarded as an extension of the PSO in a sense. Compared with the PSO, it has a better balance ability in the breadth and depth search. However, in the face of 3DP workshop scheduling problem, the iterative update of the snake group position is not as good as the crossover-mutation method of IGA.

In addition, to verify the importance of the IMM in shortening the order completion time and devices load balancing, the optimization capabilities of IGA and simple GA, PSO and SO for order completion time and device load standard deviation were compared.  Figure 6(a) shows the influence of changes in the number of 3DP devices on the completion time for the order list. The results indicated that as the number of 3DP devices increased, when the number of 3DP devices lied between two and five, the order completion time was reduced rapidly; when the number of 3DP devices lied between five and eight, the completion time of orders tends to be flat. Also, under the same number of iterations, the shortest order completion time can be achieved by IGA. It can be seen that IMM can effectively solve the problem of resource waste caused by the slow decline of the total production time of an order as the number of resources increases when the number of devices is greater than 5 and has a significant optimization effect on shortening the total production time of order. In addition, Figure 6(b) shows the changes in the overall load balance of the device with different numbers of 3DP devices. It shows that in different scenarios, the best load balancing solution can always be obtained by IGA. It can be seen that the IMM has a strong ability to optimize the load balancing between devices, which helps to improve the intelligent matching ability between devices and jobs. Combining Figures 6(a) and 6(b), it can be found that load balancing has a certain impact on order completion time. Except for IGA, when the number of devices is 5 to 6, the order completion time does not decrease but increases. At the same time, the load standard deviation between devices also increases significantly. This is because the excessive pursuit of improving the utilization rate of the devices in each job leads to poor matching results between devices and jobs. Therefore, when dealing with the M-3DP mass customization production scheduling problem, we cannot simply pursue to improve the utilization rate of equipment in each job but should look at the problem from the perspective of the overall planning and scheduling of the production workshop. To sum up, under the M-3DP mass customization production, the mismatch between devices and jobs leads to a large load standard deviation between the devices, which prolongs the total order completion time. Therefore, IMM is of great significance for M-3DP mass customization production scheduling. To a certain extent, it helps to shorten the total production time of an order, and at the same time optimize the load balancing performance among 3DP devices.

Finally, according to the multiagent intelligent collaborative scheduling method, IGA was used to solve the parallel tasks, and the task set division result, product layout, and total order completion time were calculated. For the 70 medical products, Table 5 shows the simulation results of task sets division.

Taking the task *R*_1_ as an example, the product arrangement of each job of the task *R*_1_ obtained through the product mix strategy in the IGA is shown inFigure 7.  Figure 7(a) shows the arrangement results of the projected shapes of the medical products on the processing platform, where the 450 mm × 450 mm rectangular frame represented the processing platform of the device, and each rectangle inside this platform represented a medical product to be processed, with the numbers inside indicating the product code. Figures 7(a)–7(d) represent the product arrangement results when the task *R*_1_ was divided into four jobs.

After inheriting the tasks division results, the job Agent and the 3DP device Agent are reasonably matched through the IMM embedded in the IGA. In the scenario with four sets of 3DP devices, Table 6 shows the intelligent matching results.

## 6. Conclusions and Future Work

In view of the time-consuming task and large load deviation of M-3DP large-scale customized production scheduling, a multiagent-based optimization model was established, and an IGA embedded with product mix strategy and the intelligent matching mechanism is designed to optimize production time and load balancing. Finally, numerical simulation experiments were carried out to analyze the effectiveness of the proposed method. The experimental results indicated that with a given working load and increasing device resources, IGA led to the shortest completion time, the best product arrangement, and the minimum load standard deviation of devices compared with other algorithms.

The multiagent-based M-3DP intelligent collaborative scheduling method could solve the M-3DP large-scale customized production scheduling problem under multiple materials, providing better optimization of shortening production time and balancing the load, which had certain theoretical significance. Facing the frequent occurrence of major public health events, the demand for medical products in hospitals had increased. The application of this method could shorten the production time, improve production efficiency, and alleviate the shortage of medical products to a certain extent, which had certain practical significance.

Notably, with the accelerated development of models and algorithms, emerging technologies such as the Internet of Things (IoT), artificial intelligence, and cloud computing, the M-3DP large-scale customized production scheduling method could be further improved in many aspects, including:

1. The simultaneous optimization of the three-dimensional production and the product layering direction can be considered in the model and relevant algorithms in future research, since the two-dimensional rectangle with the fixed product layer direction during the multiagent model constrains the current version of the process.
2. The current method solves the scheduling problem of minimizing production time in the same parallel machine. It is worth thinking whether future studies can develop new production scheduling methods that can adapt parallel and heterogeneous 3D printing devices simultaneously, with extended optimization objectives, such as minimizing total cost and maximizing production efficiency.
3. Emerging technologies such as IoT, blockchain, and cloud computing could be applied to deploy this method in a cloud-based environment, to promote the implementation of the industrial interconnection, build an M-3DP “smart manufacturing” supply chain, and promote the sharing and development of the resources in the medical industry [23].

## Figures and Tables

**Figure 1:** Classification of studies on 3DP allocation and scheduling problems.

**Figure 2:** M-3DP large-scale customized production scheduling simplified flow chart.

**Figure 3:** Flow chart of IGA.

**Figure 4:** Improved lowest level nesting process.

**Figure 5:** Multiagent intelligent matching mechanism.

**Figure 6:** Comparison of completion time and load balancing as 3D printing devices increase. (a) Comparison of completion time.; (b) Comparison of load balance.

**Figure 7:** Task *R*_*n*_ product arrangement result. (a) Job 1 products' arrangement. (b) Job 2 products' arrangement. (c) Job 3 products' arrangement. (d) Job 4 products' arrangement.

**Table 1:** Coding scheme.

Task 1	Product 1	Product 2	Product 3	⋯	Product *i*_1_

Task *r*	Product 1	Product 2	Product 3	⋯	Product *i*_2_

**Table 2:** Medical product information.

Medical product code	Scanning time (min)	Processing time (min)	Length (mm)	Width (mm)	Height (mm)	Printing material	Projection area (mm^2^)
1	17	266	105	101	80	1	23050
2	18	66	61	79	20	2	8552
3	6	73	30	28	22	1	5883
4	7	113	54	27	34	2	7675
5	8	70	53	143	21	2	8822
6	9	36	222	39	11	2	13660
7	14	186	36	40	56	1	7042
8	15	106	70	60	32	2	9601
9	15	170	58	58	51	1	18174
10	19	173	53	53	52	1	18306
11	20	133	40	58	40	2	7279
12	16	163	63	63	49	1	19195
13	17	156	68	68	47	1	20336
14	26	176	87	112	53	2	26139
15	28	26	79	79	8	2	11782
16	29	79	24	120	24	1	16155
17	5	140	82	58	42	2	5391
18	6	20	47	28	6	1	4122
19	22	133	148	163	40	2	12615
20	23	109	57	45	33	2	7566
21	25	66	73	91	20	1	10925
22	25	306	37	40	92	2	20352
23	26	143	57	72	43	1	11448
24	42	10	130	80	3	2	19935
25	42	213	79	59	64	2	12599
26	45	293	114	109	88	1	9179
27	34	96	27	370	29	2	15860
28	34	340	131	140	102	2	30310
29	38	266	130	70	80	2	36813
30	56	100	90	67	30	1	15879
31	60	83	150	50	25	1	18671
32	61	93	76	169	28	1	36568
33	46	316	72	104	95	2	38029
34	227	386	95	165	116	1	92067
35	247	346	73	85	104	2	71198
36	251	340	80	109	102	1	69697
37	65	340	54	125	102	2	22437
38	66	159	80	88	48	2	17500
39	71	83	140	25	145	1	42412
40	89	233	70	70	70	1	15175
41	99	200	80	121	60	1	25627
42	123	213	80	80	64	2	24460
43	130	259	77	109	78	1	25664
44	133	266	226	207	80	2	44480
45	135	133	126	137	40	1	33116
46	156	159	144	137	48	2	36814
47	159	296	89	96	89	1	61950
48	173	340	71	113	102	2	30827
49	212	406	96	87	122	2	34184
50	220	236	109	102	71	1	54796
51	339	250	203	164	75	2	48894
52	372	230	150	150	69	1	80945
53	413	66	200	200	20	1	112585
54	276	159	140	145	48	1	72909
55	598	500	161	176	150	2	102969
56	798	343	103	184	103	2	110156
57	1479	276	200	301	83	1	317492
58	284	303	86	172	91	2	93529
59	297	379	124	128	114	1	41846
60	331	233	140	151	70	1	106793
61	425	133	300	200	40	1	155674
62	477	430	123	198	129	2	86217
63	521	390	167	155	117	2	147457
64	550	416	171	171	125	1	193244
65	557	143	300	200	43	1	131703
66	598	133	280	181	40	2	145926
67	22	66	85	70	20	1	9649
68	22	90	73	79	27	2	9807
69	22	13	65	70	4	2	12248
70	1483	443	179	154	133	1	254786

**Table 3:** Algorithm parameter.

	IGA	PSO	SO

Maximum iteration	300	300	300
Population size	80	80	80
Parameter	Crossover Rate: 0.8	Cognitive weight factor *c*_1_ = 1.5	Food threshold: 0.25
	Mutation Rate: 0.1	Social weight factor *c*_2_ = 1.5	Temperature threshold: 0.6
	—	Inertia weight: 0.7	Food constant *c*_1_ = 0.5
	—	Range of speed: [−5, 5]	Exploration constant *c*_2_ = 0.05
	—	—	Development constant *c*_3_ = 2

**Table 4:** Minimum order completion time and load standard deviation of devices.

Quantity of device	IGA	PSO	SO

2	8421(0.5)	8820(2.5)	8836(40.5)
3	5717(1.88)	6067(50.5)	5869(73.8)
4	4341(3.27)	4608(71.6)	4480(85.5)
5	3552(8.25)	3711(77.3)	3588(95.2)
6	2953(10.51)	3208(173.6)	3019(34)
7	2521(23.95)	2816(136.5)	2632(58)
8	2211(7.06)	2565(251.4)	2421(244.5)

**Table 5:** Tasks division results.

Task	Job	Production time per job *C*_*mj*_ (min)

Task *R*_1_	Job *J*_1_	3738
	Job *J*_2_	1228
	Job *J*_3_	3134
	Job *J*_4_	1399

Task *R*_2_	Job *J*_5_	2132
	Job *J*_6_	970
	Job *J*_7_	2908
	Job *J*_8_	972

**Table 6:** : Intelligent matching results with four sets of 3DP devices.

3DP devices	Job	Completion time (min)	Total order completion time (min)

M1	*J*_2_, *J*_7_	4339	4341
M2	*J*_1_, *J*_4_	4333	
M3	*J*_5_, *J*_6_	4341	
M4	*J*_3_, *J*_8_	4341	

## Data Availability

The data used to support the findings of the study can be obtained from the corresponding author upon request.
